# Acute Hypersensitivity Pneumonitis Associated With a High Ki-67 Proliferative Index

**DOI:** 10.7759/cureus.7905

**Published:** 2020-04-30

**Authors:** Edward Nabrinsky, Amanda Kamar, Dereen Mohammed Saeed, Michael Pins, Arvey Stone

**Affiliations:** 1 Internal Medicine, Advocate Lutheran General Hospital, Park Ridge, USA; 2 Pathology, University of Illinois, Chicago, USA; 3 Pathology, Advocate Lutheran General Hospital, Park Ridge, USA; 4 Pulmonary and Critical Care Medicine, Advocate Lutheran General Hospital, Park Ridge, USA

**Keywords:** hypersensitivity pneumonitis, mycobacterium, mycobacterium avium complex, hsp, mac, ki-67, immunohistochemistry, proliferation

## Abstract

Hypersensitivity pneumonitis (HSP) is an interstitial lung disease caused by exposure to a large range of environmental antigens. Inhaling aerosolized particles leads to a heightened immune response. HSP comes in acute, subacute, or chronic forms, all with their own potential clinical and radiographic findings. *Mycobacterium avium* complex (MAC) is the most common nontuberculous mycobacteria and is known to cause HSP with certain exposures. However, although certain histologic findings can be seen with HSP, a high ki-67 proliferation index is unusual and more commonly associated with malignancy. In this report, we discuss a case of MAC that had acute HSP associated with a high ki-67 proliferative index.

## Introduction

Hypersensitivity pneumonitis (HSP) refers to a type of interstitial lung disease that is caused by exposure to various environmental antigens. The inhalation of aerosolized particles in occupational, domestic, or recreational environments leads to an exaggerated immune response [1]. While hundreds of different antigens are known to cause HSP, mycobacterial infections, including *Mycobacterium avium* complex (MAC), can cause this kind of presentation from both acute and chronic exposure. HSP is classified into acute, subacute, or chronic forms [2]. Even though HSP is a well-described disease, it has not been examined extensively in terms of immunohistochemical characteristics. The ki-67 proliferative index, classically associated with malignancies, has not been described in the context of HSP or bacterial infections. We report a case of acute HSP associated with MAC infection with a high ki-67 proliferative index found on immunohistochemical staining. This is the first case that we know of to have such a high elevation in ki-67 outside of malignancies.

## Case presentation

A 43-year-old male with no past medical history presented to the emergency department with eight days of fevers and cough. He reported repairing water pipes in his basement two weeks prior, but had no other environmental exposures, travel, or known sick contacts. He denied alcohol, tobacco, or illicit drug use. On presentation, his temperature was 36.5 °C, blood pressure 157/95 mmHg, pulse rate 88 bpm, respiratory rate 21 breaths/minute, and oxygen saturation 91% on room air. Leukocyte count was 7.7 cells/mm3 (normal: 4.2-11.0 cells/mm3) and procalcitonin was 0.09 ng/mL (normal: <0.10 ng/mL). Arterial blood gas was notable for partial pressure of oxygen of 67 mmHg (normal: 83-108), and two blood cultures on admission were both negative. Urine antigens for *Streptococcus pneumoniae* and *Legionella* were both negative.

A chest X-ray showed a right middle lobe infiltrate (Figure 1A). Subsequent CT pulmonary angiogram was negative for pulmonary embolism but significant for bilateral nodular and ground-glass opacities in the posterior left upper lobe, right middle lobe, and bilateral lower lobes, as well as patchy focal areas of consolidation in the right middle and left lower lobe (Figure 1B). The patient was started on ceftriaxone and doxycycline for presumed community-acquired pneumonia. He was also administered intravenous methylprednisolone due to the radiographic findings.

**Figure 1:** Imaging on presentation to the hospital A: initial chest X-ray demonstrates evidence of a right middle lobe infiltrate; B: CT pulmonary angiogram after initial chest X-ray shows evidence of bilateral ground-glass and nodular opacities (arrows), consistent with hypersensitive pneumonia CT: computed tomography

The patient would require oxygen via nasal cannula on the following hospital days, and so he underwent bronchoscopy with bronchoalveolar lavage (BAL) on hospital day three. It was notable for mucus plugging throughout the tracheobronchial tree that was purulent and thick with erythematous underlying mucosa (Figure 2). BAL was performed in the right middle lobe (Figure 3). Multiple transbronchial biopsies were also obtained.

**Figure 2:** Bronchoscopy at the level of the trachea Bronchoscopic findings demonstrate purulent and thick mucus in the setting of hypersensitivity pneumonitis

**Figure 3:** Bronchoscopy: right middle lobe of the lung Bronchoscopic finding demonstrates erythematous mucosa in the setting of hypersensitivity pneumonitis

The right lower lobe transbronchial biopsy showed marked acute and chronic inflammation of bronchial mucosa and alveoli and an aggregate of atypical epithelial cells, or cells that line organs that appear abnormal. These cells were CK7, CK5/6, and focal p40 positive (a marker often used for detection of squamous differentiation in carcinoma), as well as CD68, TTF-1, and napsin-A negative by immunohistochemical stains. A ki-67 immunohistochemical stain showed a high (85%) proliferation index, suggesting a rapidly growing lesion (Figures 4A-4D). The overall morphological features, immunoprofile, and the high proliferation index suggested squamous cell carcinoma arising in a background of squamous metaplasia. However, the absence of a mass lesion, absence of significant nuclear atypicality, presence of concomitant acute and chronic inflammation, and the benign clinical course suggested inflammatory-related, atypical squamous metaplasia of bronchial mucosa.

**Figure 4:** Various immunohistochemical stains of the transbronchial biopsies A: aggregate of atypical cells with eosinophilic cytoplasm and hyperchromatic nuclei; B: CK7 and CK5/6 immunostains show strongly positive nuclear staining in the atypical cells; C: p40 immunostain shows strongly positive nuclear staining in the atypical cells; D: Ki-67 immunostain shows a high proliferative index (85%). [H&E, original magnifications 400X (A), and 40X (B, C, D)]

Bronchoalveolar lavage results were negative for acid-fast bacilli, *Pneumocystis jirovecii* direct fluorescent antibody, and Blastomyces antigen; mycobacterial and fungal cultures and smears were pending at the time of patient discharge. Chest X-ray on the day of discharge showed improved aeration of lungs with mild residual right middle lobe airspace opacities (Figure 5A). He felt improved after five days of antibiotic therapy and went home with a steroid taper on oral prednisone after the resolution of acute HSP. The mycobacterial culture was subsequently positive for MAC, which was the presumed infectious etiology of the patient’s pneumonitis. Outpatient CT chest six weeks after discharge showed no evidence of the previously noted bilateral ground-glass densities, and there was no evidence of pulmonary scarring, fibrosis, or usual interstitial pneumonitis (Figure 5B).

**Figure 5:** Final chest X-ray on discharge and CT at follow-up A: chest X-ray on the day of discharge demonstrates mild residual right middle lobe opacity; B: follow-up chest CT six weeks after discharge demonstrates resolution of previous bilateral ground-glass and nodular opacifications, with no evidence of residual disease CT: computed tomography

## Discussion

HSP is a diffuse interstitial lung disease caused by repeated exposure to a wide spectrum of environmental antigens [1]. Because both its clinical and radiologic findings can vary, diagnosis typically depends on multiple findings rather than one singular feature. HSP tends to involve the lung parenchyma, specifically the alveoli, terminal bronchiole, and alveolar interstitium [2]. This reaction is secondary to repeated inhalation of substances to which the patient becomes sensitized [2]. Historically, most of the epidemiologic data for HSP has been from studies of farmers and bird owners; and over 300 etiologies of HSP have been documented.

High-resolution CT is primarily used for imaging over chest X-ray due to better sensitivity and specificity, which are around 75 and 90%, respectively [3]. An imaging finding that can be identified in most phases of the disease is multifocal ground-glass opacities; centrilobular nodules and evidence of air trapping can also be seen [1]. In the residual phase of the disease, findings can include honeycombing and traction bronchiectasis, both of which are associated with fibrosis and decreased rates of survival [1,4]. Other diagnostic procedures that are of benefit include BAL fluid analysis as well as lung biopsies; it is important to note that surgical lung biopsies are more sensitive than transbronchial biopsies and can show different histological findings depending on the stage of the disease [2].

In addition to environmental antigens, HSP can also be caused by antigens from microorganisms that colonize things such as air systems, water reservoirs, portable humidifiers, and hot tubs. MAC is an organism that can cause HSP in immunocompetent hosts that have a history of these kinds of exposures, particularly following hot-tube use [5]. In hot-water tubs, the agitation of water by jets of air produces aerosolization of water droplets; the combination of MAC growth and jet aerosolization predisposes to inhalation of large amounts of MAC [6]. Individuals generally respond to avoiding specific environments and do not require antibiotic therapy as part of treatment.

MAC is the most common nontuberculous mycobacteria found in isolates from respiratory specimens [7]. Pulmonary disease caused by MAC has been classified into two distinct subtypes: a more common upper lobe cavitary form and a nodular bronchiectatic form [8]. While the former has frequent cavitation, the latter occurs predominantly in non-smokers and middle-aged patients without underlying lung disease [8,9]. Radiographic findings in the nodular bronchiectatic form include bilateral interstitial or nodular change, predominantly in lower lung zones, and particularly in the right middle lobe [8]. It is interesting to note that in the nodular bronchiectatic form, isolation of MAC from sputum specimens is less consistent compared to the upper lobe cavitary form, with low numbers of organisms routinely found [8].

Histologically, findings in HSP tend to be similar regardless of the causative agent. Airway-centered distribution of interstitial inflammation is a common feature, which reflects the portal of entry for the causative agent; and if there is granulomatous involvement, it tends to resolve over time [1]. A sampling of airway cells and fluid by BAL acutely demonstrates neutrophilic infiltrate that becomes predominantly lymphocytic after 24 hours [10]. An entity known as bronchus-associated lymphoid tissue (BALT) is found in chronic HSP and maintained due to ongoing inflammation [10]. BALT has been known to express the Ki-67 antigen, which is a marker of proliferation [11]. However, the extent to which BALT tissue, or other inflammatory tissue due to HSP, can express Ki-67 is unknown and has not been widely studied.

The Ki-67 protein is strongly associated with tumor cell proliferation and is an established prognostic marker for the assessment of biopsies for patients with cancer [12]. Its prognostic value has been shown to be reliable in multiple cancers including breast, soft-tissue, lung, prostate, and cervical cancer [12,13]. Ki-67 tends to increase the more poorly differentiated a specimen becomes, and its presence has been shown to correlate with the presence of metastases and clinical staging of tumors [13]. Histologically, more than 20% of cells staining positive for Ki-67 is considered to be high in most literature, with >15% positivity having a sensitivity of >90% [14].

Aside from the chronic form of HSP mentioned previously, Ki-67 has also been detected in airway epithelial cells in the setting of interstitial pulmonary fibrosis [15]. Most of the data for Ki-67 has been in the context of malignancy, and it has not been shown to this point to have a correlation with infectious etiologies. The high amount of Ki-67 proliferation (85%) from our patient’s transbronchial biopsy has not previously been seen in the setting of a reactive airway disease. To our knowledge, this is the first case to demonstrate such a high amount of proliferation outside of a malignancy.

## Conclusions

We described a case of HSP associated with MAC infection in a middle-aged male with no predisposing conditions. Although the literature has described cases of MAC associated with HSP, our patient's disease was histologically associated with an elevated Ki-67 proliferative index, which is typically seen in aggressive malignancies. To our knowledge, this is the first case report to document this high of an elevated Ki-67 proliferative index associated with an infectious cause of HSP. Further case studies are warranted to see if other similar cases exist and if Ki-67 can be a useful immunohistochemical and prognostic marker outside of cancer.
